# Identification of the Major Molecular Types of *Cryptococcus neoformans* and *C. gattii* by Hyperbranched Rolling Circle Amplification

**DOI:** 10.1371/journal.pone.0094648

**Published:** 2014-04-15

**Authors:** Luciana Trilles, Bin Wang, Carolina Firacative, Márcia dos Santos Lazéra, Bodo Wanke, Wieland Meyer

**Affiliations:** 1 Molecular Mycology Research Laboratory, Centre for Infectious Diseases and Microbiology, Sydney Medical School – Westmead Hospital, Marie Bashir Institute for Infectious Diseases and Biosecurity, The University of Sydney, Westmead Millennium Institute for Infectious Diseases and Biosecurity, Sydney, Australia; 2 Instituto de Pesquisa Clínica Evandro Chagas, FIOCRUZ, Laboratório de Micologia, Rio de Janeiro, Brazil; 3 Westmead Millennium Institute, University of Sydney, Retroviral Genetic Laboratory, Centre for Virus Research, Sydney, Australia; Research Institute for Children and the Louisiana State University Health Sciences Center, United States of America

## Abstract

The agents of cryptococcosis *C. neoformans* and *C. gattii* are important agents of meningoencephalitis in immunocompromised and immunocompetent hosts, respectively. They are grouped into eight major molecular types, VNI-VNIV for *C. neoformans* and VGI-VGIV for *C. gattii*. These major molecular types differ in their host range, epidemiology, antifungal susceptibility and geographic distribution. To enable a rapid identification of the major molecular types and potential hybrids within the two species specific probes based on the *PLB1* gene in combination with hyperbranched rolling circle amplification (HRCA) were developed. HRCA was applied to 76 cryptococcal strains, 10 strains each representing the 7 haploid major molecular types, 4 VNIII hybrid strains and 2 inter-species hybrid strains. All strains were correctly identified to the major molecular type and or hybrid type using HRCA alone. To increase the sensitivity a semi-nested PCR step was developed, which will enable the identification of the molecular types/hybrids directly from clinical samples, harboring a low copy number of DNA (40 copies). Thus, HRCA based on the *PLB1* locus alone and in combination with a semi-nested PCR showed to be a specific and sensitive methodology, with a great potential to be used on clinical specimens for the direct diagnosis of the agents of cryptococcosis, including hybrid strains, enabling a rapid and patient tailored treatment choice of this disease.

## Introduction

Cryptococcosis is a systemic mycosis acquired by inhalation of infectious propagules (desiccated yeasts cells or spores) produced by the basidiomycetous yeasts *Cryptococcus neoformans* and *C. gattii*. Most clinical laboratories do not routinely identify the isolates to species level. However, cryptococcosis is associated with a significant morbidity and mortality and is the most common invasive fungal infection in HIV patients, with an estimated incidence of 1 million cases annually [1], mainly caused by *C. neoformans*. *C. gattii* on the other hand affects mostly immunocompetent individuals [2], [3]. Molecular epidemiological studies have identified eight major molecular types within both species. The *C. neoformans* molecular types correlate with the serotypes: VNI/AFLP1, serotype A; VNII/AFLP1A, serotype A; VNIII/AFLP3, serotype AD; and VNIV/AFLP2, serotype D. The molecular types of *C. gattii* (VG1/AFLP4; VGII/AFLP6; VGIII/AFLP5; VGIV/AFLP7) are all associated with both serotypes B and C [4].

The major molecular types of *C. neoformans* and *C. gattii* differ in their epidemiological [5], ecological characteristics, antifungal susceptibility [6], clinical presentations and therapeutic outcomes [1]. Infections caused by *C. gattii* often have a worse prognosis than those caused by *C. neoformans* [7]. The determination of the molecular types becomes important as epidemics have occur in the recent years by the molecular type VGII in the southwest of Canada and VGIII in the northwest of the USA, indicating the ability of this species to adapt to new environments [4], [8].

The currently used laboratory identification model for the agents of cryptococcosis has major limitations. *Cryptococcus* species are identified after culturing the isolates from a clinical sample followed by biochemical tests, which may delay the final diagnoses [9]. Furthermore, culture from a clinical sample is not always available, and direct examination can be imprecise, especially in the presence of atypical cells. In addition, the major molecular types within *C. neoformans* and *C. gattii* are then determined using a variety of molecular typing techniques [10], [11], [12], [13], prolonging the time of the diagnostic process.

Molecular methods have the advantage of being highly sensitive and specific to overcome the limitations of conventional diagnosis [14], [15]. Although molecular methods for the diagnosis of mycosis from clinical specimens and cultures are available, they are not yet applied in routine diagnosis laboratories [16].

In 2009, the ISHAM working group on “Genotyping *C. neoformans* and *C. gattii*” developed a consensus MultiLocus Sequence Typing (MLST) scheme for the members of the *C. neoformans/ C. gattii* species complex based on the variable regions within the capsular associated protein gene (*CAP59*), glyceraldehyde-3-phosphate dehydrogenase gene (*GPD1*), laccase (*LAC1*), phospholipase (*PLB1*), Cu, Zn superoxide dismutase (*SOD1*), orotidine monophosphate pyrophosphorylase (*URA5*) genes and intergenic spacer region (IGS1), to standardize, increase the discriminatory power and improve the inter-laboratory reproducibility of cryptococcal genotyping [13]. The generated typing results, including allele and sequence types are searchable at http://mlst.mycologylab.org.

The recently developed technique of hyperbranched rolling circle amplification (HRCA) [17] using padlock probes is a combination of a pathogen-specific molecular recognition and universal amplification. It offers an alternative method for detecting pathogens in a fast and specific way. Padlock probes are oligonucleotides of about 100 bases that contain two sequences complementary to the 5′ and 3′ end of the target sequence, joined by a genetic linker region. The hybridization with the two target regions (5′ and 3′) forms a closed, circular molecule [18] following incubation with a DNA ligase. This technique has the ability to identify single nucleotide polymorphisms (SNPs). The intensity of the signal generated by the circular molecule is increased exponentially by a hyperbranched rolling circle amplification (HRCA). Positive results can be detected by a simple electrophoresis to visualize the presence of a ladder-like pattern of dsDNA, whereas absence of bands denote negative results due to the failure of the formation of a circular molecule after probe hybridization. HRCA has been used successfully for genotyping of human populations [19], as well as viruses and bacteria [20], [21]. Recently HRCA was also used to identify the two species *C. neoformans* and *C. gattii* and to differentiate between the serotypes A and D of *C. neoformans* [22], [23].

Besides a number of available molecular identification and typing techniques, a fast, easy and highly standardized method for the identification of the major molecular types and potential hybrids within the *C. neoformans/ C. gattii* species complex is still lacking. The current study aimed to develop specific probes in combination with HRCA to identify the eight major molecular types (VNI-VNIV and VGI-VGIV) within this species complex. This methodology should allow for a fast identification of the agents, the major molecular types and hybrids involved in human and animal cryptococcosis from DNA extracts from pure cultures or directly from various clinical specimens, which will enable an informed choice of early antifungal therapy, and provide a highly sensitive tool for epidemiological surveillance.

## Materials and Methods

### Studied Isolates

Ten isolates of each of the seven haploid major molecular types of the *C. neoformans/ C. gattii* species complex, maintained at the Westmead Hospital Culture Collection, Sydney, Australia, were studied (Table 1). These strains have been chosen to represent the allelic diversity identified in the global molecular epidemiological study using the ISHAM consensus MLST scheme, maintained at mlst.mycologylab.org. In addition four VNIII hybrid isolates (VNI/VNIV) and 2 inter-species hybrid isolates VNI/VGII [24] were included in the study (Table 1), amounting to 76 strains in total. To evaluate the specificity of the HRCA probes, one strain representing each of the following common human fungal pathogens: *Candida albicans* (WM 2 = CBS 562 NT), *C. dubliniensis* (WM 602 = CBS 7987 T), *C. krusei* (WM 14 = CBS 573 T), *C. globosa* (WM 284 = CBS 599 T), *Scedosporium prolificans* (WM 06.502), *Aspergillus fumigatus* (WM 06.262), *Fusarium solani* (WM 07.291) strains were also studied. All the strains had been previously identified by routine biochemical methods and ITS sequencing and are maintained at the Westmead Hospital Culture Collection, Sydney, Australia and/or the CBS-KNAW Fungal Biodiversity Centre, Utrecht, The Netherlands.

**Table 1:** Strains tested in this study and the results obtained by HRCA.

Molecular Type by RFLP-*URA5* and ISHAM MLST scheme	Strain	Specific Probes						
		VNI	VNII	VNIV	VGI	VGII	VGIII	VGIV
VNI	WM 05.474	**+**	−	−	−	−	−	−
VNI	WM 05.524	**+**	−	−	−	−	−	−
VNI	WM 05.553	**+**	−	−	−	−	−	−
VNI	WM 05.557	**+**	−	−	−	−	−	−
VNI	WM 09.168	**+**	−	−	−	−	−	−
VNI	WM 148^S^	**+**	−	−	−	−	−	−
VNI	WM 1641	**+**	−	−	−	−	−	−
VNI	WM 1897	**+**	−	−	−	−	−	−
VNI	WM 419	**+**	−	−	−	−	−	−
VNI	WM 721	**+**	−	−	−	−	−	−
VNII	WM 05.483	−	**+**	−	−	−	−	−
VNII	WM 05.484	−	**+**	−	−	−	−	−
VNII	WM 05.485	−	**+**	−	−	−	−	−
VNII	WM 05.486	−	**+**	−	−	−	−	−
VNII	WM 05.490	−	**+**	−	−	−	−	−
VNII	WM 05.491	−	**+**	−	−	−	−	−
VNII	WM 1412	−	**+**	−	−	−	−	−
VNII	WM 1462	−	**+**	−	−	−	−	−
VNII	WM 553	−	**+**	−	−	−	−	−
VNII	WM 626^S^	−	**+**	−	−	−	−	−
VNIV	WM 01.126	−	−	**+**	−	−	−	−
VNIV	WM 02.142	−	−	**+**	−	−	−	−
VNIV	WM 04.168	−	−	**+**	−	−	−	−
VNIV	WM 04.171	−	−	**+**	−	−	−	−
VNIV	WM 04.172	−	−	**+**	−	−	−	−
VNIV	WM 04.174	−	−	**+**	−	−	−	−
VNIV	WM 05.469	−	−	**+**	−	−	−	−
VNIV	WM 1740	−	−	**+**	−	−	−	−
VNIV	WM 2242	−	−	**+**	−	−	−	−
VNIV	WM 629^S^	−	−	**+**	−	−	−	−
VNIII (VNI+VNIV)	WM 628^S^	**+**	−	**+**	−	−	−	−
VNIII (VNI+VNIV)	WM 329	**+**	−	**+**	−	−	−	−
VNIII (VNI+VNIV)	WM 1354	**+**	−	**+**	−	−	−	−
VNIII (VNI+VNIV)	WM 1738	**+**	−	**+**	−	−	−	−
VNI+VGII	WM 05.532	**+**	−	−	−	**+**	−	−
VNI+VGII	WM 05.272	**+**	−	−	−	**+**	−	−
VGI	WM 02.103	−	−	−	**+**	−	−	−
VGI	WM 05.410	−	−	−	**+**	−	−	−
VGI	WM 1218	−	−	−	**+**	−	−	−
VGI	WM 179^S^	−	−	−	**+**	−	−	−
VGI	WM 1917	−	−	−	**+**	−	−	−
VGI	WM 200	−	−	−	**+**	−	−	−
VGI	WM 2571	−	−	−	**+**	−	−	−
VGI	WM 352	−	−	−	**+**	−	−	−
VGI	WM 727	−	−	−	**+**	−	−	−
VGI	WM 834	−	−	−	**+**	−	−	−
VGII	WM 05.77	−	−	−	−	**+**	−	−
VGII	WM 06.12	−	−	−	−	**+**	−	−
VGII	WM 11.128	−	−	−	−	**+**	−	−
VGII	WM 178^S^	−	−	−	−	**+**	−	−
VGII	WM 3030	−	−	−	−	**+**	−	−
VGII	WM 1255	−	−	−	−	**+**	−	−
VGII	WM 02.32	−	−	−	−	**+**	−	−
VGII	WM 06.25	−	−	−	−	**+**	−	−
VGII	WM 05.272	−	−	−	−	**+**	−	−
VGII	WM 1008	−	−	−	−	**+**	−	−
VGIII	WM 10.121	−	−	−	−	−	**+**	−
VGIII	WM 10.17	−	−	−	−	−	**+**	−
VGIII	WM 175^S^	−	−	−	−	−	**+**	−
VGIII	WM 2088	−	−	−	−	−	**+**	−
VGIII	WM 728	−	−	−	−	−	**+**	−
VGIII*	WM 11.135	−	−	−	−	−	**+**	−
VGIII*	WM 1802	−	−	−	−	−	**+**	−
VGIII*	WM 2004	−	−	−	−	−	**+**	−
VGIII*	WM 2042	−	−	−	−	−	**+**	−
VGIII*	WM 11.32	−	−	−	−	−	**+**	−
VGIV	WM 04.20	−	−	−	−	−	−	**+**
VGIV	WM 2363	−	−	−	−	−	−	**+**
VGIV	WM 779^S^	−	−	−	−	−	−	**+**
VGIV	WM 780	−	−	−	−	−	−	**+**
VGIV	WM 05.376	−	−	−	−	−	−	**+**
VGIV	WM 08.314	−	−	−	−	−	−	**+**
VGIV	WM 1434	−	−	−	−	−	−	**+**
VGIV	WM 2567	−	−	−	−	−	−	**+**
VGIV	WM 2570	−	−	−	−	−	−	**+**
VGIV	WM 2604	−	−	−	−	−	−	**+**

**Note: +**: Positive signal with the specific probe; -: No signal with the specific probe;

*VGIII only when determined by the ISHAM MLST scheme, *URA5* RFLP is grouping them incorrectly to VGIV due to a point mutation in the RFLP restriction site; ^S^: standard strain for the major molecular type (Meyer *et al.* 2009).

### DNA Extraction and MLST Typing

DNA extractions were performed according to Ferrer *et al.* [25]. The seven MLST loci, *CAP59*, *GPD1*, *LAC1*, *SOD1*, *URA5*, *PLB1* and IGS, were amplified according to the consensus MLST scheme for *C. neoformans* and *C. gattii* [13], except for the primers used to amplify the genes *GPD1* and *LAC1* of *C. neoformans.* The *GPD1* locus of *C. neoformans* was amplified using the primers GPD1cn-F 5′ATGGTCGTCAAGGTTGGAAT 3′ and GPD1cn-R 5′ GTATTCGGCACCAGCCTCA 3′, and the *LAC1* locus of *C. neoformans* was amplified using the primers LAC1cn-F 5′ GGCGATACTATTATCGTA3′ and LAC1cn-R 5′-TTCTGGAGTGGCTAGAGC3′ [26] . Allele (AT) and sequence types (ST) were assigned according to the MLST database at http://mlst.mycologylab.org and new AT’s and ST’s were added to this database.

### Hyperbranched Rolling Circle Amplification (HRCA)

#### Amplification of the PLB gene

Amplification of the *PLB1* gene was performed in a final volume of 50 µL. Each reaction contained 50 ng of DNA, 1X PCR buffer (200 mM Tris-HCl (pH 8.4), 500 mM KCl - Invitrogen), 0.2 mM each of dATP, dCTP, dGTP, and dTTP (Invitrogen), 2 mM magnesium cloride, 1.5 U Taq DNA polymerase (Invitrogen), and 50 ng of each primer PLB1-F (5′ CTTCAGGCGGAGAGAGGTTT 3′) and PLB1-R (5′ GATTTGGCGTTG GTTTCAGT 3′) [14]. PCR was performed in a thermocycler (Perkin Elmer, California, USA) as follow: Initial denaturation at 94°C 3 min, followed by 30 cycles at 94°C 30 sec., annealing at 61°C 45 sec.; extension at 72°C 1 min; and final extension at 72°C 10 min. at 94°C [13].

#### Semi-nested PCR

To enhance the sensitivity of the target DNA detection a semi-nested PCR strategy was developed. Nested-primers with 100% homology to the *PLB1* gene of *C. neoformans* and *C. gattii* were designed (Table 2) using sequences downloaded from GeneBank (Table S1). The conditions for the semi-nested PCR were the same as the ones used for the initial *PLB1* gene amplification (see above), using 15 µl of the initial amplicon.

**Table 2:** Padlock probes and padlock probe primers.

Probesand primers	Sequence
**VNI**	5′p-TC**M** CGA GCC TCA ATG TAG GCT GAT CAt gct tct tcg gtg ccc at G CTT AGC TTG GCA TGT CAC Tcg cgc aga cac gat aGT CTA GC**K** CRA TT**R** CAG GTT GGA CAA GTT TC-3′
**VNII**	5′p-TCA GTA GAT GAA CAC ATA CAT CAT GCA GAT CAt gct tct tcg gtg ccc atA ACG ACTC CAG GTT AGC CTA Gcg cgc aga cac gat aGT CTA CCA GAG CTA TCA CGC AAA-3′
**VNIV**	5′p-GAT AAA TAA TGG GCA TAT CCT TTG C GA TCA t gct tct tcg gtg ccc at CCT ACT AGT TGC ACG CTG TTC cgc gca gac acg ata GTC TAA ACC CTG TAC TGT GGC AAC-3′
**VGI**	5′p-GCA GCA TTA ACC CAC TCA CAG GAT CAt gct tct tcg gtg ccc atC CTA GAT CAG ACG TTC CTG TCc gcg cag aca cga taG TCT ATG CAA CAA T**S**A TAA GTA TTA GGC ATA TCT TTC-3′
**VGII**	5′p-ATA CCA CCC AAC CCA GTA CTG C GA TCA t gct tct tcg gtg ccc at TAC GAG GTG CGG ATA GCT ACc gcg cag aca cga taG TCT AGC TTT CAT TCA TCA TGC TCA TA-3′
**VGIII**	5′p-GGG AGG AGT TTC GAG CCC GAT CAt gct tct tcg gtg ccc atG CTA ACC TGG TAC CGT CAT Tcg cgc aga cac gat aGT CTA CAC CAA TGA CAG GTG TCC T-3′
**VGIV**	5′p-GCT TCG GTG CTT TCA TTC ATC GAT CAt gct tct tcg gtg ccc atT CGT GGC TAG TCG AAT CTT AGc gcg cag aca cga taG TCT AC**R** GTC TCG CTT TCG GAA-3′
**RCA1**	5′-ATG GGC ACC GAA GAA GCA-3′
**RCA2**	5′-CGC GCA GAC ACG ATA-3′
**Semi-nested F**	5′ – TGG ATT AGA AAT GCC ACT GTA AG - 3′

Note: The 5′- and 3′-ends of the probes that are complementary to the target sequences are underlined. The regions where the two padlock probe-specific primers (RAC1 and RCA2) bind for real-time amplification are in lower case letters. The 5′-end of probe, p-indicates phosphorylation. Ambiguous positions were introduced according to the target sequences (in bold): M = A or C, K = G or T, R = A or G, S = C or G.

#### Padlock probe and primer design

Padlock probes were designed to target specific single nucleotide polymorphism (SNP) for each of the seven major haploid molecular types of the *C. neoformans* (VNI, VNII, and VNIV) *C. gattii* (VGI, VGII, VGIII, and VGIV). The selection of informative SNPs was based on sequences maintained in the *C. neoformans/ C. gattii* MLST database from the Molecular Mycology Laboratory, Sydney University, Australia, http://mlst.mycologylab.org, and additional sequences generated as part of the current study. The sequences used for the SNP analysis included seven unlinked genetic loci: the housekeeping genes *CAP59, GPD1, LAC1, PLB1, SOD1, URA5* and the IGS1 region. They originated from 232 *C. neoformans* (201 VNI, 20 VNII, 11 VNIV) and 359 *C. gattii* (35 VGI, 184 VGII, 126 VGIII, 14 VGIV) global strains. To identify specific SNPs for each of the seven major haploid molecular types the sequences from the 591 *C. neoformans* and *C. gattii* isolates were aligned using the program *MEGA* version 5 [27]. The specific sequence probes were designed with minimum secondary structure, as well as the 5′-end probe-binding arm Tm close to or above the ligation temperature (60°C, see below) to guarantee the effectiveness of padlock probe binding. The flanking linker region has no similarity to the respective major molecular type as defined via BlastN searches against the GenBank database. To increase 3′-end binding specificity, the 3′-end probe-binding arm was designed with Tm 10–15°C below the ligation temperature.

In addition, the primers RCA1 and RCA2 (Table 2), which are used to amplify the specific padlock probe signal during HRCA, were designed specifically to bind to the flanking linker regions of the above designed padlock probes with a Tm of about 55°C following the strategy described by Kaocharoen *et al.* [22].

#### Padlock probe ligation, exonucleolysis and signal amplification by HRCA

After amplification of the *PLB1* gene either by single or semi-nested PCR (see above), the amplicons were purified with the PureLink PCR purification kit (Invitrogen, USA). The ligation of the padlock probes to the amplified PCR products was performed according to Wang *et al.* [20], in a total reaction volume of 10 µl containing 75 ng of amplicon, 2 U of Pfu DNA ligase (Stratagene, Integrated Sciences) and 1 pmol of the padlock probe in 20 mM Tris-HCl (pH 7.5), 20 mM KCl, 10 mM MgCl_2_, 0.1% Igepal, 0.01 mMrATP, 1 mMDTT. The ligation reaction conditions included 5 min denaturation at 94°C followed by 15 cycles of 94°C for 30 s and 4 min ligation at 65°C. The ligation mixture was then subjected to exonucleolysis to remove non-circularized padlock probe and excess PCR product in order to reduce subsequent ligation-independent amplification events. The exonuclease digestion was performed in a volume of 20µl by adding 10 U of each exonucleases I and III (New England, Biolabs) to the ligation solution and incubating it at 37°C for 30 min followed by 94°C for 30 s to inactivate the exonuclease.

HRCA reactions were performed in a volume of 50 µl by adding 8 U of *Bst* DNA polymerase (New England Biolabs), 400 µM deoxynucleoside triphosphate mix, 10 pmol of each RCA primers (Table 2), 5% of dimethyl sulfoxide (v/v), and 1× SYBR Green I (Sigma-Aldrich) to the digested mixture.

Probe signals were amplified by incubation at 65°C for 30 min and the accumulation of dsDNA products was monitored in a Corbett RotorGene 3000 real-time PCR machine. Alternatively the end products could also be loaded on a 1.5% agarose gel and visualized under UV light. The positive signals are then visualized as a ladder of bands, starting at one unit circle length and extending in discrete increments to several thousands of nucleotides.

## Results

### Locus Selection

From the 7 analyzed MLST loci, the *PLB1* locus was the only one to contain specific SNPs for all 7 major haploid molecular types (Table 1), including the two most genetically related, VNI and VNII molecular types (Figure 1A). Furthermore, the *PLB1* locus has the advantage of being amplified from all molecular types using only a single primer pair. Unlike for the loci *SOD1*, *GPD1* and *LAC1*, for which different primer pairs are needed to amplify these loci form either *C. neoformans* or *C. gattii*, which would require a previous identification of both species. In addition, the IGS1 fragments are highly polymorphic and do not present specific SNPs for each major haploid molecular type. Finally the *SOD1* locus exhibited very low polymorphism among the *C. neoformans* strains, which does not allow for a differentiation amongst its major molecular types.

**Figure 1:** Association between MLST clusters and HRCA curves. (**A**) Unrooted neighbor-joining tree inferred from the combined sequences of*CAP59*, *GPD1*, *LAC1*, *SOD1*, *URA5*, *PLB1* genes and IGS of 76 strains tested in this study. Numbers on branches are bootstrap support values obtained from 1,000 pseudoreplicates. *VGIII only when determined by the ISHAM MLST scheme, *URA5* RFLP is grouping them incorrectly to VGIV due to a point mutation in the RFLP restriction site; (**B**) Amplification curves for representative strains of each major haploid molecular type, *C. neoformans* molecular types VNI, VNII and VNIV and *C. gattii* molecular types VGI, VGII, VGIII and VGIV obtained with the respective HRCA probes. (**C**) *C. neoformans/ C. gattii* VNI+VGII hybrid strain (WM 05.532), positive amplification with the HRCA probes VNI-PLB and VGII-PLB. (**D**) *C. neoformans* VNIII hybrid strain (WM 628), positive amplification with the HRCA probes VNI-PLB and VNIV-PLB. Positive results are indicated when the fluorescence signals increased exponentially.

### Primer Specificity

To demonstrate the specificity of the used primers, the *PLB1* locus [13] was also attempted to be amplified from different fungal species, including: *Candida albicans*, *C. dubliniensis*, *C. krusei*, *C. globosa*, *Scedosporium prolificans*, *Aspergillus fumigatus*, and *Fusarium solani,* commonly found in clinical specimens. No amplification was obtained from any of those species using the *PLB1* specific primers of the ISHAM *C. neoformans/ C. gattii* consensus MLST scheme (data not shown). In addition BLAST searches using the primer sequences reveal only a homology to either *C. neoformans* or *C. gattii* and did not find any matches to other basidiomycetious yeasts such as *C. laurentii, C. albidus, C. uniguttulatus* or *Trichosporon* spp.

### HRCA

HRCA amplification in combination with the detection of the generated products on a real-time-PCR was applied to ten representative strains of each major haploid molecular type (Figure 1B), as well as to 4 *C. neoformans* VNIII hybrids (Figure 1D) and 2 inter-species *C. neoformans/ C. gattii* hybrids (Figure 1C). A signal generated with the respective probes demonstrated a positive result, while no signal indicated negative results. The results of the real-time-PCR are listed in Table 1. All *C. neoformans* VNI, VNII and VNIV strains, *C. gattii* VGI, VGII, VGIII and VGIV, and the hybrid strains (VNIII and VNI/VGII) studied generated positive signals with the respective HRCA probes (Figure 1B, 1C and 1D). The probes targeting VGIII also annealed to six additional strains, which were previously identified as VGIV by *URA5*-RFLP. However, those strains showed a much closer relationship to the VGIII strains than to the VGIV in the ISHAM MLST scheme, see the phylogenetic tree in Figure 1A, represented by WM 1802, WM 2004, WM 2042 and WM 11.32. The *URA5* gene sequence analysis of those strains demonstrated one point mutation, affecting the restriction site of the enzyme *Sau96*I at the position 528 in this group of strains (WM 1802, WM 1804, WM 2004, WM 2041, WM 2042, WM 11.135), which resulted in the same fragments as the ones obtained for the major molecular type VGIV.

### Sensitivity of the Detection Method

In order to obtain the required sensitivity for a direct diagnosis of cryptococcosis from clinical or other DNA low-abundance samples, a semi-nested PCR was developed, which then was used in combination with HRCA on DNA dilutions of selected cryptococcal samples as proof of principle. When the semi-nested-F primer sequence for the *PLB1* locus was compared against the GenBank database it showed BLASTN hits with greater than 98% identity to the *C. neoformans* and *C. gattii PLB1* gene only. This demonstrated that it has a high specificity for *C. neoformans* and *C. gattii*. As such this primer was used in combination with the PLB1-R primer [13] using the PCR products from the initial *PLB1* amplification as a template to amplify a fragment of 607 bp (Table 2). The methodology then was applied on serial dilutions of DNA from *C. neoformans* and *C. gattii* cultures to determine if the sensitivity would be adequate for a possible detection directly from clinical specimens, resulting in 10 ng of DNA as the lowest limit for HRCA detection. When the semi-nested PCR strategy was applied, the sensitivity of the single copy gene detection was enhanced, enabling the detection of a minimum of 40 copies of DNA (approximately 1 pg of DNA), which is essential for the direct detection of the molecular types or species from clinical specimens (Figure 2).

**Figure 2:** Detection limit of the HRCA after semi-nested PCR. (**A**) Real-time-PCR amplification curves for the semi-nested PCR amplification of the *PLB1* locus from serial DNA dilutions of the strain WM 178 with the HRCA VGII probe. Lower curves correspond to dilutions with less than 40 copies of DNA (4×10^−1^, 4×10^−2^, 4×10^−3^, 4×10^−4^); (**B**) *PLB1* locus semi-nested PCR products from serial DNA dilutions of WM 179 strain separated on a 1.4% agarose gel.

## Discussion

Improved technologies, which accurately identify the different molecular types of *C. neoformans* and *C. gattii* or the separation of specific genotypes within those molecular types, have been increasingly important for prognostic and therapeutic implications. Despite the similar clinical features between the two species, infections caused by *C. gattii* have the tendency to induce massive inflammation and cryptococcomatas, and require additional clinical follow up. The major molecular types of *C. neoformans* (VNI-VNIV) and *C. gattii* (VGI-VGIV) are not identified in routine laboratories and the virulence of the different genotypes has not been systematically studied, although those molecular types have molecular, epidemiological, serological and antifungal susceptibility differences [28]. Similar findings have been made in connection with clinical outcomes of viral infections, which have been associated to different genotypes of the virus, as well as to genetic variations of immune genes, leading to more severe clinical manifestations [29]. Regarding fungal infections this association is unclear, but genetic variations in immune genes encoding cytokines, chemokines, and their receptors are associated with the risk for invasive mold diseases [30] and are also associated with persistent fungemia in candidemia patients [31]. Furthermore, certain MLST genotypes of *C. neoformans* were associated with a higher mortality among HIV patients in sub-Saharan Africa [32], and isolates of such genotypic group exhibited increased capsule and a more pronounced Th2 response. The same study also showed that *C. neoformans* hybrids strains were associated with increased mortality in humans, although they had attenuated virulence in mouse models [31]. All those facts together emphasize the urgent need for a differential diagnosis of the different molecular type causing human infections.

Specific padlock probes in combination with hyperbranched rolling circle amplification (HRCA) are ideal for the development of diagnostic assays, which require speed, specificity and reproducibility. The application of loop-mediated isothermal DNA amplification (LAMP) using the capsule-associated gene *CAP59* [23] was only able to identify the serotypes A and D of *C. neoformans* and *C. gattii,* but was not able to differentiate the serotypes B and C of *C. gattii*. Kaocharoen *et al.* [22] applied also HRCA to detect the major molecular types of *C. neoformans* and *C. gattii* using the internal transcribed spacer (ITS) regions of the rDNA gene cluster as a target. However, this enabled only the differentiation between VNI/VNII, VNIV and *C. gattii*. Feng *et al.* developed a duplex PCR assay using vacuolar membrane gene to differentiate between the molecular types of *C. gattii* [33], but this did not simultaneously enable the differentiation of the major molecular types of *C. neoformans*. The current study detected specific SNPs for each of the major haploid molecular types of *C. neoformans* (VNI-VNIV) and *C. gattii* (VGI-VGIV) in the *PLB1* locus, allowing for the development of specific padlock probes. HRCA using the *PLB1* locus was able to differentiate the seven major haploid molecular types of *C. neoformans* (VNI, VNII, VNIV) and *C. gattii* (VGI, VGII, VGIII, VGIV) and also identified correctly different types of hybrid isolates from DNA extracts from pure cultures.

To enable a direct detection form clinical specimens the sensitivity was increased via the development of a semi-nested PCR. This increased the detection limit to approximately 1 pg of DNA equaling a minimum of 40 copies of DNA. This brings the detection limit in the range of the DNA amounts being detected by multicopy regions, such as the ribosomal gene cluster, which is widely used as a target for the detection of fungal disease agents, where the lower detection limits range from 10 fg [34] to 500 pg [35]. However, the ribosomal regions are unable to differentiate all major molecular types within *C. neoformans* [36].

For the first time HRCA of the *PLB1* locus alone or together with the application of the herein developed semi-nested PCR approach showed to be a specific and highly sensitive methodology, with a great potential to be used on DNA extracts from pure cultures or clinical specimens for the direct identification of the different major molecular types and potential hybrids of the agents of human and animal cryptococcosis, providing the basis for a rapid and patient tailored treatment choice for this disease.

## Supporting Information

Table S1 Accession number of the sequences included in the study to design the semi-nested PCR primer.
(XLS)
